This article has been retracted.

# The Role of TAMs in Tumor Microenvironment and New Research Progress

**DOI:** 10.1155/2022/5775696

**Published:** 2022-08-15

**Authors:** Yawei Feng, Zhiqiang Ye, Furong Song, Yufeng He, Jun Liu

**Affiliations:** ^1^Department of Anesthesiology, The Third Affiliated Hospital, Sun Yat-Sen University, Guangzhou, Guangdong, China; ^2^Department of Emergency, The Third Affiliated Hospital, Sun Yat-Sen University, Guangzhou, Guangdong, China; ^3^Department of Intensive Care Medicine, The Third Affiliated Hospital, Sun Yat-Sen University, Guangzhou, Guangdong, China

## Abstract

Tumor-associated macrophages (TAMs) are an important part of tumor microenvironment (TME) and play a key role in TME, participating in the process of tumor occurrence, growth, invasion, and metastasis. Among them, metastasis to tumor tissue is the key step of malignant development of tumor. In this paper, the latest progress in the role of TAMs in the formation of tumor microenvironment is summarized. It is particularly noteworthy that cell and animal experiments show that TAMs can provide a favorable microenvironment for the occurrence and development of tumors. At the same time, clinical pathological experiments show that the accumulation of TAMs in tumor is related to poor clinical efficacy. Finally, this paper discusses the feasibility of TAMs-targeted therapy as a new indirect cancer therapy. This paper provides a theoretical basis for finding a potentially effective macrophage-targeted tumor therapy.

## 1. Introduction

Tumor microenvironment (TME) refers to the surrounding microenvironment in which tumor cells exist, including surrounding blood vessels, immune cells, fibroblasts, bone marrow-derived inflammatory cells, various signaling molecules, and extracellular matrix (ECM). Although the tumor microenvironment has a harsh environment different from that of normal tissues, the tumor microenvironment still plays a promoting role in the occurrence and development of tumors. The tumor-tumor microenvironment is often referred to as the seed-soil relationship. Tumors are closely related to the tumor microenvironment. Tumors can affect their microenvironment by releasing cell signaling molecules, promoting tumor angiogenesis, and inducing immune tolerance, while immune cells in the microenvironment can affect the growth and development of cancer cells. In a word, the tumor microenvironment is a complex integrated system formed by the interaction of tumor cells with surrounding tissues and immune cells. The existence of tumor microenvironment enhances tumor cell proliferation, migration ability, and immune evasion ability, thereby promoting the occurrence and development of tumor. In tumor microenvironment, immune cells are the main component, so inflammation is an important sign of tumor microenvironment [1]. Immune cells in tumor microenvironment interact with tumor cells, which affects the occurrence, development, and metastasis of tumors [2]. Macrophages existing in TME are called tumor-associated macrophages (TAMs) (their functions are similar to those of M2 macrophages, which can be described as M2d subtype). TAM is an important immune cell in tumor microenvironment, which mediates tumor progression by regulating tumor microenvironment [3, 4].

Macrophage is an important component of the innate immune response of the body, and it is a kind of cell group with plasticity and heterogeneity [5]. And macrophages infiltrated in tissue inflammation are derived from bone marrow monocyte precursors [6]. These precursor cells penetrate into various tissues from blood vessels and differentiate into different subtypes in different tissue microenvironments. We can roughly divide it into two categories: M1 classical activated macrophages and M2 alternative activated macrophages [7]. Interferon-*γ* (IFN-*γ*), lipopolysaccharide (LPS), and toll-like receptor (TLR) agonist can induce macrophages to differentiate into M1-type macrophages. Type M1 macrophages secrete pro-inflammatory factors such as 1(interleukin 1 (IL-1)), IL-12, IL-23, tumor necrosis factor-*α* (TNF-*α*), and CXC chemokine ligand 5 [chemokine (c-x-c motif) ligand5, CXCL9]. M1 macrophages highly express major histocompatibility complex (MHC) class I and class II molecules, which are responsible for presenting tumor-specific antigens, with high expression of IL-12 and low expression of IL-10. Therefore, M1 macrophages are an important part of inflammatory response and antitumor immunity.

On the contrary, M2 macrophages have anti-inflammatory and tumor-promoting activities. Type M2 macrophages can be further divided into four subtypes: M2a, M2b, M2c, and M2d macrophages. Th2 cytokines IL-4 and IL-13 can induce M2-type macrophages to transform into M2a-type macrophages, activation energy of TLR and immune complex can induce them to transform into M2b-type macrophages, and IL-10 can induce them to transform into M2c-type macrophages. Macrophages infiltrating into tumors are usually called tumor-associated macrophage (TAM). M2a TAM mainly mediates Th2 immune response, M2b TAM participates in humoral immunity, and M2c TAM mediates immunosuppression [8]. Type M2 macrophages secrete CC chemokine ligand 17 [chemokine (c-c motif) ligand 17, CCL17], CCL22, CCL24, etc. With low expression of IL-12 and high expression of IL-10, its tumor-killing activity is low, and TAM is closer to the functional phenotype of M2 macrophages [9, 10]. M2 TAM provides a favorable microenvironment for tumor growth and angiogenesis [11]. Clinical studies have confirmed that the infiltration of TAM is negatively correlated with the overall survival rate of tumor patients. Ding et al. [12] found that M1 macrophages can inhibit the growth of tumors and improve the treatment results of glioma patients; the ratio of M2 cells is related to tumor proliferation and poor prognosis. Macrophage phenotype can be used as a potential biomarker to evaluate the malignant degree, invasion, and prognosis of tumor. This review reviewed the relationship between TAMs and TME, including the concept of ATMs, an overview of the tumor microenvironment, the association of TAMs and tumor microenvironment, TAMs and tumor immunosuppression, TAMs promoting drug resistance in tumor cells, and the role of TAMs in tumor therapy, thus providing a theoretical basis for finding a potentially effective macrophage-targeted tumor treatment.

## 2. TAMs

### 2.1. The Origin of TAMs

Macrophages in tissues were originally thought to originate from bone marrow. However, local self-sustaining alveolar and abdominal macrophages, Kupffer cells, epidermal Langerhans cells, and brain microglia from the original yolk sac precursor are called tissue-resident macrophages. Although there is evidence that all kinds of macrophages can coexist in tumors, the recruited macrophages account for the majority of TAMs. At present, it is impossible to evaluate the respective roles of these macrophages in different tumor stages, and further research is still needed. Bone marrow-derived peripheral blood mononuclear cells (PBMCs) were recruited to the local tumor and further differentiated into TAMs under the action of chemokines secreted by stromal cells and tumor cells in the tumor microenvironment. Whether macrophages come from yolk sac or bone marrow, CSF1 is the main regulator and chemokine of most macrophages [13]. The combination of CCL2 and its receptor CCR2 directly mediates the recruitment of monocytes into primary and metastatic tumors [14]. In the animal model of human breast cancer, CCL18 binds to its receptor PITPNM3 and mediates the recruitment of macrophages in cooperation with CSF2 [15]. In the colon cancer model, it was found that the recruitment of macrophages was mediated by the binding of CCL20 to its receptor CCR6, and the absence of this chemokine led to the down-regulation of monocytes and/or TAMs and the regression of tumors [16]. CXCL12/CXCR4 axis mediates the accumulation of TAMs and is related to the progression of B16 malignant melanoma [17].

### 2.2. Polarization and Typing of TAMs

Macrophages are derived from marrow cell lines, yolk sacs, embryonic precursors of fetal liver progenitor cells, or monocyte precursors of hematopoietic origin, and have good proliferation ability [18, 19]. According to the mirror nomenclature, macrophages can be divided into two categories, and the two extremes of functional state spectrum: (1) Under the stimulation of IFN-*γ* (interferon-*γ*) [20], LPS (lipopolysaccharide), and TNF-*α* (tumor necrosis factor-*α*), they can differentiate into classic activated macrophages (M1 phenotype). M1 macrophages produce inflammatory and immunostimulating cytokines, trigger adaptive response, secrete reactive oxygen species (ROS) and nitrogen intermediates, participate in the innate defense of the host, and have cytotoxic effects on transformed cells. They are mainly involved in Th1-type immune response, resist pathogen invasion, and monitor tumor lesions, so they are regarded as antitumor or “good” macrophages. (2) Under the induction of interleukin (IL-4, IL-10, and IL-13) secreted by helper T cell 2, it differentiated into replacement activated macrophages (M2 phenotype) [21, 22]. M2 phenotype plays an important role in humoral immunity, wound healing, and tissue remodeling mediated by helper T cells 2 [21]. In addition, the M2 type produces growth factors, activates tissue repair and angiogenesis, has high-resolution inactivation activity, and can suppress adaptive immune responses, and is therefore considered a “bad” macrophage that promotes tumors [23]. M2 phenotype can be subdivided into three subgroups: M2a, M2b, and M2c. M2a macrophages are triggered by IL-4 or IL-13, M2b macrophages are polarized by toll-like receptor (TLR) and IL-1Ra, and M2c macrophages are subjected to IL-10, transforming growth factor-*β* (TGF-*β*). Based on extensive research, it has been proposed that TAMs in tumor microenvironment (TME) are multi-polarized as anti-inflammatory macrophages (M2 phenotype), which not only can promote tumor angiogenesis, growth, and the expression of various immunosuppressive cytokines but also has the potential to enhance the activities of IL-10, TGF-*β*, and hyperuricase-1 and stimulate the expression of cell surface markers [24, 25]. This is contrary to the function of most pro-inflammatory mediators including TNF-*α*, IL-1b, and IL-12 secreted by M1 macrophages [26].

TAMs can be composed of different subgroups and have different functions in tumor areas. In the pathological examination of gastric cancer patients, TAMs mainly distributed in the following: (1) around the cancer nest (especially in the mucosa); (2) around the necrotic focus of cancer tissue; and (3) perivascular and fibrous stroma of cancer tissue [27]. TAMs participate in tumor progression by regulating the expression of chemokines, growth factors, and scavenger receptors, and tumor cells regulate TAMs polarization by releasing various cytokines. Scavenger receptors CD163 and CD206, as cell surface markers, are highly expressed in M2 TAMs and are considered to be useful for distinguishing M2 phenotype from other M1 phenotype macrophages [28, 29]. Notch signal transduction pathway, as a highly conservative signal transduction pathway, involves many cell biological processes including proliferation, angiogenesis, hypoxia, tumor stem cell activity, and epithelial-mesenchymal transformation (EMT), and can also be involved in inducing TAMs polarization [30–32]. The ligand of TLR (such as LPS or IFN-*γ*) can induce macrophages to polarize into M1 phenotype, promote inflammatory reaction, and kill tumor cells. Cytokines (such as IL-4 or IL-13) of 2(T helper 2 (Th2)) can stimulate macrophages to transform into M2 phenotype, inhibit inflammatory response, and promote tumor progression [33]. In addition, inhibition of Akt/mTOR pathway can induce macrophages to polarize towards M1 type. On the contrary, activation of Akt/mTOR pathway can lead to M2 polarization, thus inhibiting the secretion of pro-inflammatory factors. In the tumor microenvironment, various transcription factors, such as IRF-4, Stat6, PPAR-*γ*, endothelin-2, VEGF-A, and EMAPII, can regulate the substitution of activated M2 macrophages [34]. The phenotype of TAMs is tunable at the stage of tumor progression, similar to M1 in the early stages and M2 in the late stages. In addition, TAMs increase the degradation of the extracellular matrix and basement membrane primarily by promoting tumor invasion because it does not produce substances that promote tumor cell proliferation.

It can be seen that the infiltration degree of TAMs is closely related to tumor progress.

## 3. Overview of Tumor Microenvironment

TME refers to the extracellular environment on which the survival of tumor cells depends, including immune cells such as lymphocytes infiltrated in the tumor, myeloid-derived inflammatory cells, vascular system composed of endothelial cells, and supporting components such as extracellular matrix (ECM) and fibroblasts that play a supporting role, as well as various signal molecules that connect various cellular components in the microenvironment. Tumor microenvironment (TME) is an important part of tumor. The understanding of the essence of TME in cancer evolution has led to the change from the cancer development concept centered on tumor cells to the concept of complex tumor ecosystem supporting tumor growth, metastasis, and spread. TME has a strong immunosuppressive effect, which is also a key reason why the clinical efficacy of most cancer treatments that stimulate the immune response of immune cells to fight cancer is limited.

## 4. TAMs and Tumor Microenvironment

Tumor microenvironment is formed by a variety of cells, various chemical factors, cytokines, enzymes, and extracellular matrix [35, 36]. The association between tumor and TME begins at its early growth stage and exists in the whole development process. TME's contribution to tumor progression largely depends on “residents” who have settled down. Heterogeneous cells in TME are crucial to the initial formation of tumor. It represents most stromal cells in CAF TME, which can secrete collagen and cytokines, helping to form the structural framework of extracellular matrix [37, 38]. Extracellular matrix has been proved to be an independent risk factor for lymph node metastasis in early gastric cancer [39]. Myeloid inhibitory cell (MDSC) is a variety of bone marrow progenitor cells, which can produce 1(arginase 1 (ARG1)) to promote tumor cell growth and inhibit immune cell function. Activated T cells and Treg cell subsets can express cytotoxic T lymphocyte associated protein 4 (CTLA-4, CD152) on the cell surface. This protein can be used as an immune checkpoint molecule, down-regulate T cells, and inhibit antitumor response [40]. TAMs can promote tumorigenesis through the following ways: (1) releasing many angiogenesis factors, including vascular endothelial growth factor (VEGF), platelet-derived growth factor (PDGF), and basic fibroblast growth factor (bFGF), which stimulate angiogenesis in tumors; (2) TAMs secretes many signal molecules, growth factors, and matrix metalloproteinase (MMP), thus activating epithelial-mesenchymal transformation, invasion, and metastasis of tumor cells; (3) TAMs contributes to the high-level expression of IL-10 and TGF-*β* in TME and also expresses some low-level inflammatory cytokines (such as IL-1, IL-6, IL-12, and TNF-*α*). In response to the stimulation from TME, TAMs promote the formation and maintenance of tumor stem cells through various cytokines. (4) TAMs negatively regulate cytotoxic effector cells, such as CD8+, NK, and NKT cells and promote the expansion of immunosuppressive Treg cells and MDSC through the interaction of cytokines and metabolic enzymes with surface receptors.

As a member of TME, the biological activity of TAMs will be affected by various chemicals in TME. LPS, IFN-*γ*, and GMCSF act through transcription factors Stat1, IRF1, or IRF5 to induce the production of pro-inflammatory factors, inducible nitric oxide synthase, and antitumor cytokines and chemokines and stimulate the activation of M1 TAMs [41]. Tumor-derived IL-4, IL-13, IL-10, M-CSF, and lactic acid activate arginase-dependent arginine metabolism and promote the activation of M2 TAMs through the action of transcription factors Stat3/6, Klf2/4, and IRF3/5 [42–44]. Inhibition of non-receptor tyrosine kinase FAK in TME will reduce the recruitment and migration of CAF, which is the key regulator of macrophage migration [45]. Qi Zou [46] found that the expression of tumor suppressor gene VPS33B was negatively correlated with macrophage immune infiltration, and it could reduce the expression of ANXA2 to regulate the chemokine pathway, thus regulating the chemotactic level of TAMs in TME and affecting the prognosis of patients. Wu Hao [47] confirmed that by knocking down the expression of LncRNA NR028, the function of M2 macrophages in promoting gastric cancer cell metastasis was weakened. In addition, it was found that B- and T-lymphocyte attenuator (BTLA) was positively correlated with the expression of macrophages. Blocking BTLA can significantly block the inhibition of T cell proliferation by macrophages [48]. In addition, blocking PD-L1 can significantly block the inhibition of T cell proliferation by mononuclear phagocytes. Zhang Yanqing et al. [49] found that TGF-*β*1 down-regulated the expression of miR-155, and macrophages tended to be activated in M2 type. On the other hand, the down-regulation of miR-155 could increase the expression of TGFBRII.ii. and enhance the regulatory effect of TGF-*β*1 on macrophages. According to related reports, signal pathways such as Stat3, Wnt, and NF-*κ*B are also involved in the regulation of tumor microenvironment, affecting tumor progression [50, 51], and the specific mechanism remains to be confirmed.

## 5. TAMs Are Involved in the Occurrence and Development of Tumors

TAMs play an extremely important role in the occurrence and development of tumors. Firstly, TAMs promote tumor angiogenesis and provide nutrition for tumor growth. Secondly, TAMs can promote the invasion and migration of tumor cells by degrading ECM. Before tumor metastasis, macrophages are recruited to distant organs and secrete some cell molecules to gradually change the microenvironment of the metastatic tissues, so as to prepare a suitable microenvironment for distant metastasis and early survival of tumor cells, that is, pre-metastatic niche. In addition, macrophages secrete some immunosuppressive factors such as transforming growth factor *β* (TGF-*β*) and IL-10 to inhibit tumor immunity. Other data showed that TAMs-derived IL-6 promoted the development of liver cancer through STAT3 signaling pathway, and TAMs-derived IL-10 promoted the development of non-small cell lung cancer through STAT1 signaling pathway. These results reveal that tumor-infiltrating macrophages play an important role in the occurrence and development of cancer.

### 5.1. The Formation of Immune Suppression Microenvironment

TAMs are the main immunomodulatory cell in TME, which is involved in inhibiting the antitumor effect of cytotoxic T lymphocytes. In malignant pleural effusion, the secretion of TGF-*β* by TAMs increased, which led to the decrease of antitumor effect of T cells. In the mouse tumor model, TAMs inhibited the proliferation of CD8+T cells, and to some extent, induced the production of ROS by iNOS or Arginase I, leading to immunosuppression. IL-10 produced by TAMs can induce the expression of costimulatory molecule PD-L1 in monocytes, thus inhibiting the antitumor effect of cytotoxic T lymphocytes. In addition, PGE2, IL-10, and indoleamine 2,3-dioxygenase from TAMs play an important role in the induction of regulatory T cells (Tregs). CCL17, CCL18, and CCL22 from TAMs are important chemokines of Tregs, and Tregs further inhibit the immune effect of T cells in TME.

### 5.2. TAMs Promote Tumor Metastasis and the Establishment of TME

The mechanism of TAMs promoting tumor progression also includes enhancing tumor metastasis and establishing pre-metastasis microenvironment. In the model of human transplanted tumor, it was found that CCL18 derived from TAMs promoted the invasion and metastasis of tumor cells. The migration of tumor cells through ECM is necessary for tumor metastasis, and TAMs are believed to promote the migration and invasion of tumor cells through ECM. TAMs can produce proteases, including cathepsin B, MMP2, MMP7, and MMP9, and can cleave ECM, providing a channel and pathway for tumor cell metastasis.

Epithelial-mesenchymal transition (EMT) plays an important role in tumor progression and metastasis. Therefore, clarifying the regulatory mechanism of EMT will greatly improve our understanding of tumor migration and invasion. More and more evidence shows that EMT is an important feature of tumor changes after the interaction between TAMs and tumor cells, and related factors derived from TAMs play an important role in the occurrence and development of EMT. According to the research results of animal models, TAMs play a key role in the microenvironment before tumor formation and metastasis. TNF-*α*, VEGF, and TGF-*β* secreted by TAMs in tumor tissues can be transported to the target organs through blood flow, inducing local macrophages to produce S100A8 and serum amyloid A3. These factors further recruit macrophages and tumor cells into the target organs and promote the formation of metastatic foci. Therefore, TAMs are considered to affect not only the local microenvironment but also the macrophages of the whole body, thus leading to the progress of the tumor.

### 5.3. TAMs Promote Tumor Angiogenesis

TAMs play an important role in tumorigenesis and development and play an important role in angiogenesis. In 1971, Judah Folkman [52] proposed that tumor growth depends on angiogenesis, that is, the sprouting of new blood vessels from existing capillaries, which are the supply and removal of oxygen and nutrients, thereby promoting tumor growth, proliferation, invasion, and transfer. Zeisberger et al. [53] used chlorophosphate liposome to specifically remove macrophages, which could obviously inhibit tumor growth and angiogenesis. Therefore, TAMs are involved in tumor angiogenesis and play an important role.

TAMs can promote angiogenesis by secreting various angiogenic factors, such as VEGF, PDGF, transforming growth factor-*β* (TGF-*β*), tumor necrosis factor-*α* (TNF-*α*), IL-1*β*, IL-8, C-C chemokine ligand 2 (CCL2), C-X-C chemokine ligand 8 (Cx8), and C-X-C chemokine ligand 12 (CXCL12), and the ability of angiogenesis depends on the number of these growth factors and the density of blood vessels, and the density of microvessels is closely related to the density of TAMs. Studies have shown that TAMs can promote angiogenesis by promoting matrix formation and releasing PDGF. Thymidine phosphorylase, an angiogenic factor secreted by TAMs, can promote endothelial cell migration and participate in angiogenesis, and its expression level is related to tumor angiogenesis [54]. TAMs can also secrete enzymes that contribute to angiogenesis, such as MMP2, MMP7, MMP9, MMP12, and 2(cyclooxygenase 2 (COX2)). In addition, TAMs can promote coagulation activity through fibrin deposition, thus indirectly promoting angiogenesis.

Due to the vigorous metabolism and rapid growth of tumor cells, but poor development of the vascular system, hypoxia is a common feature of most solid tumors. It is one of the signs of hypoxia TME. In order to help tumor cells overcome nutritional deficiency and transform TME into a more suitable environment for tumor cells to survive, cells perceive and balance hypoxia level through transcription of many genes [55]. TAMs in the hypoxic region of tumor prefer to stay at the hypoxic site, which can induce the secretion of hypoxia-inducible factor (HIF) and enhance the angiogenesis ability of tumor cells. TAMs in hypoxic tumor area are closely related to the increase of VEGFA expression [56]. HIF is composed of HIF-1*α*, HIF-2*α*, and HIF-1*β*. Under normal oxygen conditions, the target gene of HIF-1 is turned off, and proline hydroxylase (PHD) can detect the oxygen content in cells and respond to the existence of oxygen by hydroxylating HIF-1*α* subunits on proline residues. HIF-1*α* produces binding sites on proline 402 and 531 residues, and HIF-2*α* produces binding sites on proline 405 and 531 residues. Under hypoxia, TAMs began to express a large number of transcription factors such as HIF, but the hydroxylation of proline to HIF-1*α* was weakened and the degradation of HIF-1*α* was blocked due to the damage of PHD activity. Non-hydroxylated HIF-1*α* is more stable than hydroxylated HIF-1*α*, resulting in increased expression of protein. This protein can then interact with HIF-1*β* and promote the transcription of HIF-1 target gene, and promote angiogenesis by activating the transcription of angiogenesis factor VEGF, thus increasing the invasion ability of tumor cells [56]. 1(neuropilin 1 (NRP1)) is the receptor of signal 3a (SEMA3A), which is related to the signal response of TAMs in hypoxia. If NRP1 is knocked out, it can restore antitumor immunity and inhibit angiogenesis. Once macrophages enter the hypoxic site, the expression of NRP1 in TAMs is down-regulated, which leads to the decrease of TAMs redistribution, inhibition of tumor growth, and reduction of angiogenesis. Badawi et al. [57] found that in colon cancer, the number of TAMs infiltration in malignant/invasive tumors was significantly higher than that in benign polyps, thus increasing the blood vessel density. It can be seen that the infiltration of TAMs is closely related to angiogenesis of colon cancer cells and is positively related to blood vessel density. The same phenomenon has also been reported in oral squamous cell carcinoma, gastric cancer, breast cancer, and pancreatic neuroendocrine tumor [58–61].

### 5.4. TME Role of TAMs in TME in Self-Renewal of Tumor Stem Cells

Cancer stem cells (CSCs) represent a group of cancer cells with self-renewal ability and can produce malignant offspring tumors. Because CSCs are resistant to chemotherapy drugs, it also becomes the key to control tumor recurrence [62]. It has been reported that TAMs can control the self-renewal ability and drug resistance of CSCs through the complex network of cytokines, chemokines, growth factors, and extracellular matrix molecules. Yi et al. [63] found that glioma-derived cells can produce higher levels of CCL2, CCL5, VEGF-*α*, and neurotensin than glioma cells, which indicates that CSCs play an important role in the recruitment of TAMs by secreting macrophage chemokines. Another study also proposed the multiple roles of TAMs in CSCs self-renewal through the paracrine circulation mode of epidermal growth factor signaling pathway. As Yang et al. [64] suggested in the report, in mouse breast cancer cells, TAMs can promote the phosphorylation of STAT3 by activating EGF signal and induce SOX-2 expression that maintains CSCs phenotype of tumor cells. Matrix components in TME can also regulate the function of TAMs in assisting CSCs in self-renewal. As Okuda et al. mentioned in the report, hyaluronic acid produced from metastatic breast CSCs promotes the interaction between TAMs and CSCs, and then TAMs secrete platelet-derived growth factor (PDGF) BB to activate fibroblasts. However, osteoblasts can induce the expression of fibroblast growth factors (FGF) 7 and 9, assist CSCs in self-renewal, and improve the ability of tumor invasion and metastasis to bone microenvironment [65].

## 6. TAMs and Tumor Immunosuppression

The formation of immunosuppressive microenvironment is one of the immune escape mechanisms. Tumor immunosuppressive microenvironment is mainly composed of immunosuppressive molecules, matrix components, inhibitory immune cells, and related immunosuppressive cytokines. Among them, immunosuppressive cells mainly include TAMs, regulatory T cells, MDSC, and cancer-related CAF, which play a powerful role in tumorigenesis. Regulatory T lymphocytes (Tregs) can induce apoptosis, cytolysis, and local immune tolerance of effector cells and play a role in autoimmune, cancer, and metabolic inflammation [66–68]. MDSC can interfere with innate immune function and inhibit immune cell response [69, 70]. Cancer-related CAF not only stimulates the proliferation of tumor cells but also regulates the function of immune cells in tumors and mediates inflammation [71].

Macrophages are induced by TGF-*β* to differentiate into M2-type expression, namely, TAMs [72], which simultaneously inhibit the proliferation of CD4+ T cells and prevent T cells from attacking tumor cells; at the same time, it secretes growth factors to nourish tumor cells and promote tumor tissue angiogenesis [69]. IL-10 is an effective immunosuppressive cytokine related to cancer. The secretion of TGF-*α* and IL-10 by TAMs can induce the expression of programmed death protein ligand, so as to inhibit the killing of tumor by T cells [73]. In addition, they also inhibit the migration of natural killer cells and inhibit the immune response by reducing the function of NK cells [74]. Studies have found that vasoactive intestinal peptide up-regulates the expression level of SIRP*α* gene and protein in activated macrophages, competitively inhibits the activation of NF-*κ*B and PI3K-AKT signals, and negatively regulates the immune function of macrophages [75]. PD-1 is a member of the immunoglobulin superfamily and is an important immunosuppressive molecule. Among 100 gastric adenocarcinoma patients collected by Xie Jun, the expression of B7-H1 was as high as 65% [76]. As a ligand, the interaction with PD-1 significantly inhibited the function of effector T cells and was involved in the immunosuppressive process.

## 7. TAMs Affect TME and Promote Drug Resistance of Tumor Cells

Drug resistance is often an inevitable obstacle to the long-term effectiveness of clinical cancer chemotherapy drugs. In TME, the depletion or inhibition of TAMs can reduce the drug resistance of chemotherapy and radiotherapy in vivo and in vitro. Studies have shown [77, 78] that IL-6 cytokine produced by TAMs blocks the expression of tumor suppressor miR-204-5p by activating IL-6R/activator of transcription 3(STAT3) pathway in colon cancer cells, and miR-204-5p is a functional target that mediates TAMs-induced chemotherapy resistance in colon cancer. In addition, Yin et al. [79] showed that miR-155-5p in TAMs was frequently down-regulated, which led to the increase of the expression of the transcription factor CCAAT enhancer binding protein (C/EBP) *β*, while the transcription of C/EBP*β* in TAMs could activate IL-6, and then IL-6 induced the chemotherapy resistance of tumor cells by activating the IL6R/STAT3/miR204-5P pathway.

## 8. The Role of TAMs in Tumor Therapy

TAMs promote tumor growth in different tumor models, and the increase of TAMs number is closely related to the poor prognosis of various tumors. Pathological sections of 20 ovarian cancer specimens with complete clinical data showed that there were significant differences in lymph node metastasis and staging of ovarian cancer by the International Federation of Gynecology and Obstetrics (FIGO) between the high expression group and the low expression group of TAMs specific molecular marker CD68 [80]. Wan Ting et al. [81] found that the infiltration density of TAMs in ovarian cancer tissue was higher than that in benign lesions, and the 5-year survival rate was significantly lower than that of patients with low-density invasive cancer of TAMs. Studies on patients with locally advanced breast cancer found that the high expression group of CD68 was more sensitive to chemotherapy, and the short-term curative effect was better, but the long-term prognosis was not satisfactory [82]. Jiang Nan et al. [83] also confirmed that TAMs are an independent risk factor for poor prognosis of breast cancer. It was found that the 5-year survival rate of gastric cancer with high TAMs density in the nest was high, while the 5-year survival rate was low with high TAMs density in the cancer stroma [84]. Hou Lin and Wang Xin-jian [85] show that the patients with high TAMs count have poor prognosis of gastric cancer. Ishigami et al. [86] used immunohistochemical method and anti-CD68 antibody to evaluate the invasion of TAMs in 97 patients with gastric cancer. It was found that the surgical prognosis of high TAMs count group was significantly worse than that of low count group, and TAMs invasion could be used as a prognostic marker of gastric cancer.

The main treatment strategies of tumor are surgical resection, chemotherapy, and immunotherapy. Surgical resection has strict indications, which are not applicable to most advanced patients. At present, the exploration of tumor immunotherapy is getting deeper and deeper, and monoclonal antibodies, cytokines, cytotoxic cells, T cell infusion, and gene transfer vaccines have been applied in practice. TAMs are related to TME. As a driving factor of tumor progression, TAMs are a potential therapeutic target. Targeted therapy for TAMs includes the following directions.

### 8.1. Blocking the Recruitment of Macrophages

In recent years, it has become a new antitumor treatment strategy to eliminate TAMs by inhibiting the recruitment of macrophages.

CCL2 and CCR2 are important players in macrophage recruitment. Blocking of the CCL2/CCR2 signaling pathway significantly reduces TAMs in tumors, thereby inhibiting tumor growth, invasion, metastasis, and angiogenesis. Teng et al. found that the recruitment of inflammatory monocytes, infiltration, and polarization of TAM can be inhibited by knocking out CCR2 or applying CCR2 antagonist, thus inhibiting tumor growth and prolonging the survival time of liver cancer mice [87]. In addition, similar CCR2 inhibitors, such as CCX872-B, BMS-813160, PF-04136309, and MLN1202, have also shown efficacy in mouse models and have now entered the clinical trial stage [88]. However, it should be noted that a study based on breast cancer model shows that stopping the blocking of CCL2/CCR2 signal pathway may aggravate the progression and metastasis of the tumor, thus aggravating the condition [89].

Colony stimulating factor 1 (CSF1)/CSF1R signaling pathway is also an important participant in the survival, recruitment, and differentiation of macrophages. TAM stimulates the aggregation and movement of macrophages in tumors by secreting CSF1. After CSF1 is combined with its receptor CSF1R, it can promote the survival and differentiation of human monocytes into macrophages, increase the infiltration of TAM, and promote the growth, invasion, metastasis, and angiogenesis of tumors [90]. At present, some CSF1R inhibitors have been developed, such as Pexidartinib (PLX3397), BLZ945, ARRY-382, PXL7486, JNJ-40346527, IMC-CS4, MCS110, PD-0360324, Cabiralizumab, Emactuzumab, and AMG820.

### 8.2. Activation of Targeted TAMs

Targeting TAMs activation with different strategies is also an effective method for tumor treatment. CSF1/CSF1R signaling pathway plays a key role in the production of bone marrow mononuclear cells and TAMs polarization in tumor tissues. Therefore, CSF1/CSF1R signaling pathway is a promising target for cancer therapy. Animal model studies have found that CSF1 gene deletion can significantly reduce the metastasis of breast cancer and neuroendocrine tumor and delay tumor progression [91]. Based on the above results, a number of clinical trials of CSF1/CSF1R inhibitors have been completed or are under way.

Macrophage surface markers can be used as effective therapeutic targets. Mannose receptor CD206 can be regarded as a specific target of macrophages. Single-chain peptide bound to CD206 receptor is linked to nanocarrier and selectively targets CD206+TAMs [92]. Legumain is a stress protein, which belongs to asparagine endopeptidase family. It is overexpressed in TAMs and can be used as an effective therapeutic target [93]. Immunotoxin-binding monoclonal antibody targeting scavenger receptor A and CD52 on macrophage surface has been studied in ovarian cancer [94]. In addition, the clinical trial of alemtuzumab (anti-CD52 antibody) in the treatment of tumor is underway.

Trabectedin (ET743, Yondelis) reduces the number of TAMs in tumor tissues by inducing the apoptosis of monocytes and macrophages [95, 96]. At present, trabectedin has obtained the marketing approval of the European Commission for the treatment of ovarian cancer and soft tissue sarcoma and was approved by FDA in 2015 for the treatment of unresectable metastatic liposarcoma or leiomyosarcoma [97].

### 8.3. Depletion of TAMs

Many studies have confirmed that the density of TAMs in tumor tissues is related to poor prognosis. The higher the density, the faster the tumor grows. Therefore, the depletion of TAMs already existing in TME is an effective way to inhibit tumor growth. Early studies [98] found that bisphosphonates can clear monocytes and macrophages. At present, the most in-depth study of depleted TAMs is the inhibition of CSF-1/CSF-1R signal axis. As mentioned above, many strategies have been developed to interfere with this macrophage survival pathway, including monoclonal antibodies against small molecule inhibitors of CSF-1 or CSF-1R. The results show that [99] CSF-1R is expressed on TAMs in tumor microenvironment, and CSF-1R inhibitor may exhaust M2 macrophages in tumor microenvironment. Emactuzumab is a monoclonal antibody against CSF-1R, and its combination with immunotherapy drugs has been used in clinical trials of NSCLC. The depletion of TAMs can also be achieved by targeting surface molecules, including CD52, scavenger receptor A (SR-A), folate receptor *β* (FR-*β*), and CD206 [100]. Intervention on these targets can exhaust tumor-promoting macrophages, thus inhibiting angiogenesis and delaying tumor progression, which may have a certain prospect in preventing tumor progression.

### 8.4. Reprogramming of TAMs

As mentioned earlier, one of the key characteristics of macrophages is their plasticity, which allows them to change their phenotype according to different tumor microenvironments. Therefore, reprogramming TAMs into antitumor phenotypes is a very potential tumor treatment strategy. Antitumor macrophages (M1 type) have a good ability to clear and destroy tumor cells [101]. Our previous research results show that Pseudomonas aeruginosa can polarize CD163+TAMs into M1 macrophages during the treatment of malignant pleural effusion, suggesting that reprogramming CD163+TAMs can be a potential treatment strategy for malignant pleural effusion [102].

At present, nanoparticles are gradually used to polarize TAMs into antitumor phenotype. Zanganeh et al. [103] found that nanometer ferric oxide (ferumoxytol) could significantly inhibit the growth of mouse subcutaneous adenocarcinoma, accompanied by the increase of M1 macrophages in tumor tissues. Manganese dioxide nanoparticles can enhance the chemotherapy response by inducing TAMs to polarize into M1 macrophages [104]. IL-12-loaded nanoparticles can reverse the antitumor function of macrophages [105].

CD40 is a marker on the surface of macrophages. The combination of CD40 agonist and gemcitabine was used to treat unresectable pancreatic cancer. It was found that this method could promote tumor regression by enhancing the function of antitumor macrophages [106]. ChiLob7/4 is a chimeric CD40 monoclonal antibody, which can induce the production of pro-inflammatory cytokines in macrophages. The results of a phase I clinical trial study on CD40-expressing solid tumors and diffuse large B lymphoma which are resistant to conventional therapy show that this therapy has broad application prospects [107]. Other clinical trials targeting CD40 molecule are currently underway.

TLR agonist, anti-CD40 antibody, and IL-10 antibody were used to activate NF-*κ*B signal pathway, and polarized TAMs showed antitumor phenotype [108]. A small molecule inhibitor of STAT3 (WP1066) can reverse the immune tolerance of malignant glioma patients, selectively induce the expression of costimulatory molecules CD80, CD86, and IL-12 in peripheral blood and tumor-infiltrated macrophages, and induce macrophages to polarize to antitumor phenotype [109]. At present, a clinical trial is studying the treatment of recurrent malignant glioma and metastasis with this drug.

Thymosin-*α* is an immunomodulatory hormone, which can retrain TAMs into dendritic cells, produce high levels of pro-inflammatory cytokines, and participate in antitumor immune response. In addition, some clinical trials have confirmed that Thymosin-*α* can prolong the survival of patients with metastatic melanoma and advanced non-small cell lung cancer [110].

*β*-glucan is a polysaccharide from yeast, which can polarize TAMs into M1 macrophages, and is a powerful antitumor immunomodulator [111]. In a phase II clinical trial, the application of *β*-glucan polymer (PGG) showed appropriate antitumor activity [112].

## 9. Summary

In the tumor microenvironment, the recruitment and polarization of TAMs and immunosuppression in tumors can affect tumor recurrence, metastasis, and drug resistance. At present, there are many clinical studies to improve the survival rate of tumor patients through the intervention of TAMs. By in-depth study of the role of TAMs in the tumor microenvironment, we can further understand the interaction between the tumor microenvironment and tumor cells, find more effective macrophage-targeted therapy, and interact with cytotoxicity, target or immune checkpoint combined with blocking therapy. More and more effective new antitumor drugs will be developed in the future. With the increasing development of tumor microenvironment research, more efficient tumor treatment methods and drugs will come out in the near future.

## Data Availability

The experimental data used to support the findings of this study are available from the corresponding author upon request.
